# The Effect of Chemotherapy Induction Therapy on the Pancreas in Patients with Acute Lymphoblastic Leukemia

**DOI:** 10.1155/2022/4978456

**Published:** 2022-08-02

**Authors:** Temesgen Gebeyehu Wondmeneh, Ayal Tsegaye Mekonnen

**Affiliations:** ^1^Department of Public Health, College of Health Science, Samara University, Ethiopia; ^2^Department of Biomedical, College of Health Science, Samara University, Ethiopia

## Abstract

**Background:**

The effect of chemotherapy induction on the pancreatic in patients with acute lymphoblastic leukemia is not described in Ethiopia. The study determined the chemotherapy drug-induced pancreatitis in patients with acute lymphoblastic leukemia.

**Method:**

A preexperimental study (pretest and posttests) was conducted in forty patients with acute lymphoblastic leukemia. For some skewed data, a log transformation was computed. The back transformation was then calculated. Descriptive statistics and a mixed-model ANOVA were used to analyze the data. A post hoc Bonferroni test was used. A *p* value < 0.05 was declared statistically significant.

**Results:**

In this study, no clinically significant acute pancreatitis occurred. Elevated amylase and lipase levels, indicating grade 2 acute pancreatitis, were observed in 25% and 17.5% of patients, respectively. Amylase enzyme levels in children differed significantly from preinduction to the second week of induction (*p* = 0.001) and fourth week of induction (*p* = 0.001), as well as between the second and fourth weeks of induction (*p* = 0.033), but adults' amylase enzyme levels did not differ significantly (*p* = 0.2). Lipase levels in adults are nearly identical in all three measures, implying that there is no statistically significant difference (*p* = 0.775). However, the level of lipase enzyme in children was significantly higher from baseline to two and four weeks of induction (*p* = 0.007) but not between two and four weeks of induction (*p* = 0.129).

**Conclusion:**

Clinically significant acute pancreatitis did not occur, but patients experienced mild (grade 2) acute pancreatitis. Amylase and lipase enzymes responded significantly to chemotherapy induction in children. Chemotherapy drugs should be given without altering pancreatic enzymes, specifically in children.

## 1. Background

Acute pancreatitis is the most common clinical disease. It is a condition of varying degrees of severity, with some patients having mild, self-limited attacks, and others experiencing severe, morbid, and usually fatal attacks [1–3]. Amylase and lipase levels are generally high during acute pancreatitis [4]. In a WHO database, 525 different drugs that can induce acute pancreatitis as an adverse reaction are listed [5]. The prevalence of drug-induced pancreatitis is still unclear because most incidences have been documented only as a single case reports [6]. The occurrence of drug-induced acute pancreatitis is generally rare; however, the disease is associated with significant morbidity and mortality, making early identification of the causative agent critical [7, 8]. A significant number of drugs regularly used for gastrointestinal diseases were found to be the causes of acute pancreatitis. The etiology and pathophysiology of drug-induced pancreatitis are unknown [9]. Although remarkable progress has been made in the treatment of children with acute lymphoblastic leukemia in many low- and middle-income countries (LMIC), survival rates remain much lower than in high-income countries. Inadequate supportive care and excess mortality from toxicity are major reasons for treatment failure in children with acute lymphoblastic leukemia in low-income countries [10]. The incidence of acute pancreatitis was 8.4% in patients receiving chemotherapy induction in the United States [11], 11% in patients treated with COG regimens in California [12], 1.1% in patients who received vincristine plus L-asparaginase in Mexico [13], and 8.3% in Thailand [14]. In Egypt, 7.31% of patients who received the pediatric DFCP regimen developed acute pancreatitis. Adolescents and young adults were more toxic than children [15]. Patients aged 10 to 18 years were more likely to experience asparaginase-related pancreatitis than those younger than 10 years [16, 17]. Pancreatitis risk factors were genetics, older age, and a higher cumulative doses of asparaginase [18, 19]. The cumulative doses of L-asparaginase had no effect on pancreatitis [20–22]. Early detection and identification of risk groups or risk factors for chemotherapy-induced pancreatitis is desirable for the management and monitoring of patients, but it is not yet available in Ethiopia. Thus, this study determines chemotherapy-induced pancreatitis and its associated factors in patients with acute lymphoblastic leukemia in Ethiopia.

## 2. Materials and Methods

### 2.1. Study Area

The study was conducted at Black Lion Hospital in Addis Ababa, Ethiopia. It is the largest public referral hospital among tertiary institutions in the country where patients from all over the country receive referral services.

### 2.2. Patient Information

Patients aged 2 to 52 years who were newly diagnosed with acute lymphoblastic leukemia at Black Lion Hospital between July 1 and September 30, 2019, were included. The same study group is divided into three groups based on the dosages of induction chemotherapy drugs. These were the baseline study group, the second week induction study group, and the fourth week induction study group.

Eligible criteria: patients have been in the hospital for at least one month but have not yet begun induction therapy and patients who have never experienced pancreatitis

Study design and sample size: a preexperimental (pretest and posttest) study design was used to assess chemotherapy-induced acute pancreatitis. Each of the three groups involved 40 patients with acute lymphoblastic leukemia, for a total of 120. The study participants were selected using a purposive sampling method

Ethical considerations: ethical clearance was obtained from the ethical review committee of Addis Ababa University's College of Health Science. All methods were performed in accordance with the relevant guidelines and regulations. The study did not harm anyone who participated in the research. Informed written consent was obtained from all adults and the parents or legal guardians of all participants who were under 18 years of age. In addition to parental informed written consent, the child's informed written consent was obtained as much as the child's ability. The right of participants to withdraw at any time is respected. By eliminating any identifier from questionnaires, confidentiality was preserved. Before receiving informed written consent, investigators read and explained the consent form and gave them the opportunity to ask questions. The investigators then responded to the questions. After being briefed about the study, participants freely agreed to participate and signed the consent form

### 2.3. Measurements of Amylase and Lipase Enzymes Were as Follows

The pancreatic function test is a laboratory test used to measure levels of amylase and lipase enzyme at baseline, fifteen, and thirty-day induction. The normal levels of amylase and lipase are 28–100 IU/L and 16–63 IU/L, respectively, based on leaflet Roche-COBAS Integra®400-chemistry laboratory analyzer.

#### 2.3.1. Variables and Operational Definitions

Dependent variable is acute pancreatitis.

Independent variables were age, sex, weight, alcohol intake, blood transfusion, and induction chemotherapy drugs.

Induction protocol is as follows: all patients were treated in accordance with Modified Berlin-Frankfurt-Munster dose schedule in phase A induction chemotherapy [23] (Table 1).

In this study, acute pancreatitis was defined by the presence of two criteria, which were abdominal pain (acute onset of a persistent, severe, and epigastric pain often radiating to the back) and serum amylase and/or lipase levels that were at least three times the upper limit of normal [24, 25].

The Common Toxicity Criteria for Adverse Events (CTCAE) version 5.0 is used to grade the severity of acute pancreatitis [26] (Table 2).

A single dash (-) indicates that a definition is not available.

Underweight: it is considered when the body mass index (BMI) is below the fifth percentile [27].

Pediatric age (children): according to Black Lion Hospital's service provision, patients aged 15 years or younger at the time of diagnosis or treatment are admitted to the pediatric ward.

#### 2.3.2. Data Collection and Sampling Procedures

After brief clarification, informed consent was obtained from all study participants. This was followed by structured interview questionnaires to gather background information. The induction period lasted a month and serum blood samples were taken once before and twice after chemotherapy.

#### 2.3.3. Blood Sample Data Collection and Processing

Blood samples were taken from participants in 5 mL serum separator tubes once before induction (baseline) and twice after chemotherapy induction (after the second and fourth weeks). The specimen was allowed to clot for 20 minutes. The specimen was centrifuged at 1500 rpm for 5 minutes, and the serum was separated and stored at 4°C until an assay was performed. The pancreatic function test was analyzed from serum at the Ethiopian Public Health Institute (Roche-COBAS Integra® 400) clinical chemistry laboratory.

#### 2.3.4. Test Analysis

The pancreatic function test included measurement of the concentration of amylase and lipase serum. The analysis was performed using the principle of a spectrophotometer to measure the absorption spectrum of the analyst at every wavelength. The automatic chemistry analyzer was a Roche-COBAS Integra® 400. All tests were performed based on the manufacturer's protocol.

#### 2.3.5. Preanalytical Phase

To maintain the quality of the blood sample, the standard operating procedures were followed in all steps of specimen collection. Processing samples were kept at 2–8°C until they were analyzed at the Black Lion Specialized Hospital. Blood samples with incomplete information were rejected.

#### 2.3.6. Analytical Phase

Quality control (percicontrolclinical chemistry level one with 25025400 lot number and level two with 34827300 lot number) was checked before running patient samples to test the performance of clinical chemistry analyzers.

#### 2.3.7. Data Quality Assurance

There was a fair procedure for the selection of study participants and outcome measurements.

### 2.4. Data Analysis

The data were entered into SPSS version twenty-three database sheets and checked for completeness. The Shapiro-Wilk test revealed that the baseline amylase, baseline lipase, and fourth week lipase distributions were skewed. These skewed pancreatic function tests were transformed using the log 10 transformation. A back transformation is then performed for each value. Proportion, mean, and standard deviation were computed. A mixed-model ANOVA was used to determine the association between independent factors and the dependent variable. Greenhouse-Geisser was used to correct the findings when the assumption of sphericity was violated. When the F-test was significant, a post hoc Bonferroni test was used. The *p* value < 0.05 was used to determine statistically significant.

## 3. Results

### 3.1. Sociodemographic Characteristics of Patients with Acute Lymphoblastic Leukemia

Forty patients with acute lymphoblastic leukemia were measured three times a month. Fifty-five percent of those were men. Forty-five percent were between the ages of 1 and 10 years. The median age was 14 years (range: 2–52 years). More than 85% of participants were transfused with blood during the 4-week study period. About 17.5% of patients with acute lymphocytic leukemia were underweight. Approximately 13% of adult patients were alcoholic drinkers (Table 3).

### 3.2. The Occurrence and Severity of Chemotherapy-Induced Acute Pancreatitis in Patients with Acute Lymphoblastic Leukemia

No patients had met the criteria for acute pancreatitis. Therefore, chemotherapy-induced acute pancreatitis did not occur in any patients. However, there was grade 2 pancreatitis, as seen by comparable higher amylase levels in the second and fourth week induction groups (25%). About 17.5% of patients had elevated lipase levels, indicating grade 2 pancreatitis in the 4-week induction group. Other grades of pancreatitis were not observed (Table 4).

### 3.3. The Effects of Induction Chemotherapy Drugs on the Amylase Enzyme in Patients with Acute Lymphoblastic Leukemia

In each of the three subsequent measurements, a total of 40 similar patients with acute lymphoblastic leukemia participated. Study subjects were followed up for one month. Mauchly's sphericity test revealed that the sphericity hypothesis was violated (*p* = 0.024). As a result, a Greenhouse-Geisser correction (*ɛ* = 0.85) was used. There was an interaction between the three groups (baseline, second, and fourth week) and age groups (pediatric and adult age) (*F* (1.69, 64.2) = 3.58, *p* = 0.033), but no interaction between the three groups and the other resting variables (sex, weight, blood transfusion, and alcoholic drinker) (*p* > 0.05). Thus, the effect of chemotherapy induction on amylase levels differs between adults and children. The effect of chemotherapy induction on amylase enzyme levels in adults and children is very comparable from baseline to the second week induction period, but after two weeks of induction, the effect of chemotherapy induction in adults is constant, whereas, in children, the effect of chemotherapy induction on amylase continuously increases dramatically. Children's amylase enzyme levels differed significantly from preinduction to the second and fourth weeks of induction, as well as between the second and fourth weeks of induction (*F* (1.3, 25) = 14.9, *p* = 0.001), but adults' amylase enzyme levels did not differ significantly (*F* (1.45, 27.53) = 1.8, *p* = 0.2) (Table 5). The interaction nature of chemotherapeutic induction on the amylase enzyme in children and adults are depicted in Figure 1.

### 3.4. The Effect of Induction Chemotherapeutic Drugs on the Lipase Enzyme in Patients with Acute Lymphoblastic Leukemia

Mauchly's sphericity test indicates that the condition of sphericity was not met (*p* = 0.001). The Greenhouse-Geisser correction was thus used to adjust the violation of sphericity (*ɛ* = 0.77). The effect of induction with chemotherapy drugs on lipase enzyme is different between adults and children (*F* (1.54, 58.54) = 4.471, *p* = 0.023), indicating that the effect of induction with chemotherapy drugs on lipase enzyme is age-dependent. Lipase levels in adults are nearly identical in all three measures (baseline, second week of induction and fourth week of induction), implying that there is no statistically significant difference (*F* (1.4, 26.8) = 0.162, *p* = 0.775). However, the level of lipase enzyme in children elevated from baseline to postinduction is statistically significant (*F* (1.26, 24) = 8.94, *p* = 0.004) (Table 6).  Figure 2 depicts the nature of the relationship between induction chemotherapeutic agents and lipase levels in adults and children.

## 4. Discussion

Three consecutive measurements were taken for a month in a similar study group. The study was a preliminary investigation of the effects of induction chemotherapeutic medications on pancreas in Ethiopia. In our study, no patients had chemotherapy drug-induced acute pancreatitis. This finding contradicts prior studies from other countries [11–15], which found acute pancreatitis despite its rarity. The differences between the present finding and the prior studies may be due to sampling size, the health status of patients, standard care of hospitals, the type of chemotherapy drug regimen, and short-term follow-up. Genetic variation could be another significant difference [18, 19]. The absence of acute pancreatitis in this study's sample size suggests that it is rare even with a larger sample size, which is consistent with earlier findings [7, 8]. Although clinically significant acute pancreatitis did not occur, a significant proportion of patients experienced grade 2 acute pancreatitis. This finding revealed that chemotherapeutic drug exposure caused minimal, temporary, and reversible pancreatic cell injury. This evidence supports previous findings that acute pancreatitis severity ranges from mild to severe and is self-limiting [1–4]. The effect of chemotherapy drugs on pancreatic function tests differed between children and adults, and this difference was age-dependent. Amylase enzyme levels increased significantly in children from baseline to 4 weeks of induction, but not in adults. Similarly, the lipase levels in adults remained almost identical during the chemotherapeutic induction phase. However, lipase levels in children increased dramatically from baseline to postinduction. These findings indicated that children receiving chemotherapy drugs were more toxic and susceptible to pancreatitis than adults. The evidence is consistent with earlier findings [15–19]. Children's mean amylase and lipase enzyme levels increased as chemotherapy drug dosages increased from baseline to 4-week induction. This suggests that cumulative chemotherapeutic drug dosages may have increased the risk of developing pancreatitis. This evidence is in line with earlier studies [18, 19], despite contradicting other earlier studies [20–22].

Applying a mixed-model ANOVA is useful in determining the association or interaction between independent variables and a dependent variable, as well as in identifying risky age groups. Measuring a similar group three times and comparing the results of these three groups avoided variation between the groups. Clinicians will benefit from this study because they will gain a better understanding of the transient and reversible effects of chemotherapy drugs on the pancreas. Future research should use a large sample size and a long follow-up period to identify the chemotherapeutic drugs that cause pancreatitis.

## 5. Conclusion

Clinically significant acute pancreatitis did not occur, but patients experienced grade 2 acute pancreatitis. Chemotherapy drug induction temporarily elevates children's pancreatic enzymes (amylase and lipase) and is related to cumulative chemotherapeutic drug dosages. In adults, the amylase and lipase enzymes did not respond significantly to chemotherapy induction. Chemotherapy drugs should be given without altering pancreatic enzymes, particularly in children, and patients should be closely monitored.

## Figures and Tables

**Figure 1:** The effects of chemotherapy induction on amylase levels in adults and pediatrics.

**Figure 2:** The effect of chemotherapy induction on lipase levels in adults and pediatrics.

**Table 1:** Modified Berlin-Frankfurt-Munster 95 dose schedule in phase A induction chemotherapy.

Duration	Drugs	Dose	Route of administration	Days
4 weeks	Prednisone	60 mg/m^2^/day	Oral	Days 1-28
	Vincristine	1.5 mg/m^2^/dose	IV	Days 1, 8, 15, 22
	Doxorubicin	30 mg/m^2^/dose	IV	Days 1, 8, 15, 22
	L-asparaginase	5000 IU/m^2^	IM	Days 8, 14, 21, 27

**Table 2:** Grading pancreatitis severity using CTCAE version 5.0.

Grading	Pancreatitis remarkers
Grade 1	—
Grade 2	Enzyme elevation; radiologic finding only
Grade 3	Sever pain, vomiting, medical intervention indicated
Grade 4	Life threatening
Grade 5	Death

**Table 3:** Sociodemographic characteristics of patients with acute lymphoblastic leukemia at Black Lion Hospital.

Number of acute leukemia patients = 40			
Variables	Categorized variables	No of patients	%
Sex	Males	22	55
	Females	18	45
Pediatrics age (in year)	1-5	9	22.5
	5-10	9	22.5
	10-15	4	10
Adults age (in years)	15-20	5	12.5
	20-25	3	7.5
	25-30	7	17.5
	>30	3	7.5
Underweight	Yes	7	17.5
	No	33	82.5
Blood transfusion	Yes	35	87.5
	No	5	12.5
Alcohol drinking	Yes	5	12.5
	No	35	87.5

**Table 4:** Pancreatitis grading using the Common Toxicity Criteria for Adverse Events (CTCAE) version 5.0.

Pancreas function tests	Measurement time	Patients with grading 2 pancreatitis No. (%)
Elevated amylase	After second week induction	10 (25)
	After fourth week induction	10 (25)
Elevated lipase	After second week induction	1 (2.5)
	After fourth week induction	7 (17.5%)

**Table 5:** The mean of amylase enzyme before and after chemotherapy induction for adults and pediatrics.

Age group	Measurement time Mean ± S.D	Measurement time Mean ± S.D	p-value
Pediatrics or children	Preinduction 59.4 IU/L ± 26.6 IU/L	After two-week induction 74.7 IU/L ± 28.1 IU/L	0.001
		After 4-week induction 94.9 IU/L ± 33.5 IU/L	0.001
	After 2-week induction 74.7 IU/L ± 28.1 IU/L	After 4-week induction 94.9 IU/L ± 33.5 IU/L	0.033
Adults	Preinduction	67.74 IU/L ± 21.51 IU/L	0.2
	After 2-week induction	79.5 IU/L ± 38.5 IU/L	
	After 4-week induction	79.4 IU/L ± 38.6 IU/L	

S.D = standard deviation.

**Table 6:** The mean lipase levels in adults and children before and after chemotherapy medication induction.

Age group	Measurement time Mean ± S.D	Measurement time Mean ± S.D	*p* value
Pediatrics or children	Preinduction 23.5 IU/L ± 9.8 IU/L	After 2-week induction 31.1 IU/L ± 14.4 IU/L	0.007
		After 4-week induction 42.2 IU/L ± 23.7 IU/L	0.007
	After 2-week induction 31.1 IU/L ± 14.4 IU/L	After 4-week induction 42.2 IU/L ± 23.7 IU/L	0.129
Adults	Preinduction	36.8 IU/L ± 18.8 IU/L	0.775
	After 2-week induction	34.1 IU/L ± 18.9 IU/L	
	After 4-week induction	35.8 IU/L ± 18.5 IU/L	

S.D = standard deviation.

## Data Availability

The data set used to analyze and support the findings of this study is available from the corresponding author upon request.

## Abbreviations

ANOVA: Analysis of variance
SPSS: Statically Package for Social Science.
